The article "Improved Support Vector Machine based on CNN-SVD for vision-threatening diabetic retinopathy detection and classification" was retracted in 2025. Reasons: original data or images not available; concerns about the data; concerns about the peer review; concerns about the citations.

# Improved Support Vector Machine based on CNN-SVD for vision-threatening diabetic retinopathy detection and classification

**DOI:** 10.1371/journal.pone.0295951

**Published:** 2024-01-02

**Authors:** Anas Bilal, Azhar Imran, Talha Imtiaz Baig, Xiaowen Liu, Haixia Long, Abdulkareem Alzahrani, Muhammad Shafiq

**Affiliations:** 1 College of Information Science and Technology, Hainan Normal University, Haikou, 571158, China; 2 Department of Creative Technologies, Air University, Islamabad, Pakistan; 3 School of Life Science and Technology, University of Electronic Science and Technology of China UESTC, Chengdu, Sichuan, China; 4 School of Science and Technology, University of Management and Technology UMT, Lahore, Punjab, Pakistan; 5 Faculty of Computer Science & Information Technology, Al Baha University, Al Baha, Saudi Arabia; 6 School of Information Engineering, Qujing Normal University, Sichuan, China; University of Manitoba, CANADA

## Abstract

The integration of artificial intelligence (AI) in diagnosing diabetic retinopathy, a major contributor to global vision impairment, is becoming increasingly pronounced. Notably, the detection of vision-threatening diabetic retinopathy (VTDR) has been significantly fortified through automated techniques. Traditionally, the reliance on manual analysis of retinal images, albeit slow and error-prone, constituted the conventional approach. Addressing this, our study introduces a novel methodology that amplifies the robustness and precision of the detection process. This is complemented by the groundbreaking Hierarchical Block Attention (HBA) and HBA-U-Net architecture, which notably propel attention mechanisms in image segmentation. This innovative model refines image processing without imposing excessive computational demands by honing in on individual pixel intricacies, spatial relationships, and channel-specific attention. Building upon this innovation, our proposed method employs a multi-stage strategy encompassing data pre-processing, feature extraction via a hybrid CNN-SVD model, and classification employing an amalgamation of Improved Support Vector Machine-Radial Basis Function (ISVM-RBF), DT, and KNN techniques. Rigorously tested on the IDRiD dataset classified into five severity tiers, the hybrid model yields remarkable performance, achieving a 99.18% accuracy, 98.15% sensitivity, and 100% specificity in VTDR detection, thus surpassing existing methods. These results underscore a more potent avenue for diagnosing and addressing this crucial ocular condition while underscoring AI’s transformative potential in medical care, particularly in ophthalmology.

## Introduction

As one of the most complex sensory organs in humans, the eye plays a crucial role in our ability to perceive objects, colors, and depths. It consists of several components: the retina, iris, pupil, optic nerve, and lens. Disorders in any of these parts can have severe consequences, ranging from visual impairment to blindness. Among the numerous eye disorders, four prevalent ones often result in vision loss or blindness: Age-related Macular Degeneration (AMD) [1], Glaucoma [2], Cataracts [3], and Diabetic Retinopathy (DR) [4].

AMD, a retinal disease affecting central vision, damages the macula and is the primary cause of vision loss in individuals over 60. Diabetic retinopathy, on the other hand, is characterized by ongoing damage to the retina’s blood vessels due to persistent high blood sugar levels. A specific form of this condition, vision-threatening diabetic retinopathy (VTDR), ranks as the second most common retinal disease that can lead to blurred vision or blindness. The number of DR patients is projected to reach approximately 439 million by 2030, making it the leading cause of blindness and visual impairment among the working-age population globally [5,6].

VTDR’s microvascular damage includes microaneurysms, hemorrhages, and exudates. Fig 1 illustrates various kinds of damage, such as a microaneurysm appearing as a dot, a hemorrhage resembling a circular blot, and cotton wool spots that result from nerve fiber swelling. These abnormalities, including microaneurysms (MAs), hemorrhages (HEs), hard exudates (HEXUs), and soft exudates (SEXUs), are closely linked to DR, and each indicates the disease’s severity in a patient [7,8].

**Fig 1:** FIs with different severity of VTDR.

VTDR can be categorized into five severity stages: normal, mild, moderate, severe, and proliferative, as shown in Fig 2. Different lesions characterize the first four stages, while specific symptoms like retinal neovascularization mark the fifth stage [9–12].

**Fig 2:** A DR fundus image shows early signs of VTDR, soft exudates, microaneurysms, hard exudates, and hemorrhage.

Detecting VTDR early is essential, especially since early warning signs are often absent, and damage to blood vessels is irreversible. Identifying VTDR manually is time-consuming, requiring expert clinicians to analyze digital color images of the retina’s fundus. The required skills and equipment are often lacking in areas with large diabetes populations, making diagnosis even more challenging.To overcome these challenges, researchers have been working on automated DR detection using computer-aided diagnostic (CAD)-based methods. Several machine learning algorithms, image processing, and data mining approaches have been suggested to classify DR’s early diagnosis and severity level. Although the applied CAD methods have been familiar and beneficial, they still present significant challenges in the medical field [13–16].

### Research gaps and motivation

In diabetic retinopathy (DR) detection, a significant research gap revolves around the challenges in automation, efficiency, and accuracy. Though various methodologies employing machine learning and deep learning, including convolutional neural networks (CNNs), have emerged, several challenges persist:

- Existing methods often consume extensive resources, limiting their applicability.
- Some current methodologies are hindered by a lack of accuracy, particularly in complex scenarios.
- The availability of varied datasets to develop well-rounded models remains constrained.
- Traditional methods often lean on manual feature extraction, resulting in potential errors and inefficiency.

Our research is motivated by the desire to fill these gaps and develop a method that improves the detection accuracy of VTDR while minimizing computational costs and errors.

### Solution and findings

Our study approached these challenges with a comprehensive methodology involving pre-processing, data augmentation, feature extraction, and classification stages tailored to VTDR detection. Our principal findings and contributions include the following:

- This study proposed the Hierarchical Block Attention (HBA) block and HBA-U-Net architecture. Integrating content, relative position, and channel attention mechanisms elevates accuracy without drastically increasing computational complexity.
- A novel Improved Support Vector Machine (ISVM) combined with distinct models based on a majority voting approach. This innovative technique decreases error proneness, resulting in more reliable outcomes.
- Utilizing a hybrid CNN-SVD model, this study successfully extracted essential features from fundus images after pre-processing and data augmentation. Our method reduced the features to a more manageable number, enhancing the model’s simplicity and effectiveness.
- Our proposed model was tested on the IDRID datasets containing 516 retinal fundus images, leading to promising results. The methodology exhibited strong capabilities in identifying early signs of disease and discerning healthy eyes, demonstrating its potential in real-world applications.
- The calculated accuracy, sensitivity, specificity, f1-score, and computational time revealed the enhanced diagnostic ability of our model compared to previous approaches.
- By reducing reliance on manual feature extraction and increasing efficiency and accuracy, our research has significant implications for the global struggle against visual impairment and blindness caused by VTDR.
- The significance of our research lies in its potential to revolutionize VTDR detection. Addressing identified gaps and leveraging innovative techniques has laid the groundwork for a more accurate, efficient, and broadly applicable solution to one of the leading causes of visual impairment worldwide. The insights gleaned from our study serve as a foundation for future research and practical applications in the ongoing battle against VTDR. The rest of this paper is organized as follows: "The ’Literature Review’ section comprehensively examines previous studies and relevant literature. The ’Materials and Methods’ section describes the research methodology employed. The findings and associated discussions are covered in the ’Results and Discussion’ section. Finally, the ’Conclusion’ section offers insights and observations related to the proposed work, encapsulating the study’s overall implications.

## Literature review

Diabetic retinopathy (DR) detection has witnessed significant advancements in recent years, driven by applying various deep learning and machine learning models. Recognizing the critical role of early and accurate diagnosis in managing and treating DR, researchers have endeavored to develop computational models that identify DR lesions and classify them according to severity. This literature review delves into recent studies, revealing a landscape of innovation and persistent challenges. It offers a comprehensive view of the methodologies, findings, and limitations of the field’s current state.

There have been several new methods for locating retinal structures developed recently. To achieve reliable localization of the Optic Disc (OD), for instance, an encoder-decoder network incorporating a deep residual structure and recursive learning technique has been developed. The next step is a region-based convolutional neural network (R-CNN) technique that is end-to-end and intended to segment the optic disc and cup simultaneously [17,18]. Similarly, several studies have used convolutional neural network (CNN) models to locate the fovea precisely. Even though the fovea and OD have a strong spatial association, very little research has focused on segmenting these structures together [19,20].

Furthermore, models developed on healthy eyes often show poor generalization when used on sick eyes with retinal abnormalities. A noteworthy example is in [21], where a modified version of U-Net++ with an EfficientNet encoder showed state-of-the-art (SOTA) outcomes in landmark identification for diseases like AMD and glaucoma. However, there is untapped potential in combining attention processes with convolutional backbone networks to highlight retinal abnormalities important for landmark identification in degraded retinal settings.

Automated diabetic retinopathy (DR) classification through various innovative methods. One approach used MobileNetv2, achieving an 87.40\% accuracy rate [22]. Another implemented a Deep Learning Multi-Label Feature Extraction model with pre-processing and transfer learning, showing its potential for large-scale DR screening [23]. A novel method combining patch division and deep-feature engineering with DenseNet201 outperformed prior methods, illustrating its efficacy in enhancing DR detection accuracy [24].

Continuing from this focus on retinal structure detection, The study by Reference [25] employed the ResNet50 and VGG16 architectures to detect DR lesions, notable for computational robustness but struggled with potential inaccuracy in identifying microaneurysms. Another research [26] utilized five distinct CNN architectures to categorize DR lesions by severity, though burdened by high computational costs.

Deep learning was harnessed by Reference [27] to predict DR class, achieving impressive specificity and sensitivity values but hinting at possible enhancement needs. Inception V3 to create a Siamese-like CNN architecture for DR detection, with some concerns regarding efficacy with matched fundus photos.

The DeepDR framework [28] introduced specificity and sensitivity values of 97.7% and 97.5% for DR detection, suggesting further testing on more complex datasets. An SVM hybrid model by Reference [29] achieved remarkable sensitivity, accuracy, and specificity, proposing deep learning for future comparison.

Utilizing a U-Net and transfer learning, Reference [30] segmented and classified DR with state-of-the-art performance, hinting at future refinements. The study in Reference [31] leveraged morphological, geometrical, and orientational properties for DR classification and recognized the need for detection accuracy improvement.

Research by Reference [32] applied optimization methods with SVM to achieve 96.91% accuracy, looking to high-performance technologies in future work. Reference [33] used thresholding and regularized regression methods for DR risk prediction, calling for enhancement in detection performance. Texture characteristics and SVM in Reference [34] detected high-risk DR with 86% accuracy but noted a limited dataset. Lastly, a two-stage CNNs approach by Reference [35] identified retinal areas of interest but faced computational challenges.

A recent study employed the extreme learning machine (ELM) approach to address diabetic retinopathy (DR) using a novel method for classification. Through pre-processing and utilizing a hybrid neural network model, the proposed system achieved accuracy rates of 99.73% for binary classification and up to 98.09% for five-stage DR classification. This approach surpasses existing methods, highlighting its efficiency in DR diagnosis [36].

The reviewed literature, including the innovative ELM-based approach, illuminates a panorama of diverse and sophisticated DR detection and classification methodologies. From leveraging various CNN architectures to applying hybrid models, the field demonstrates a blend of successes and challenges. Computational cost, dataset limitations, accuracy enhancement, and early-stage diagnosis are recurring themes across these studies. In contrast, our proposed methodology addresses many identified gaps by utilizing a hybrid CNN-SVD model for feature extraction and an improved SVM-RBF with DT and KNN for classification. By integrating pre-processing, data augmentation, and specific stages designed for VTDR detection, our approach aims to offer a more accurate and efficient solution. Unlike the reviewed methods that often rely on manual feature extraction or other classifiers, our methodology reduces errors. It demonstrates its novelty in providing a tailored solution for DR diagnosis, even identifying early signs of disease. Our findings and approaches contribute to the ongoing effort to improve the diagnosis of this leading cause of visual impairment and blindness worldwide, situating our work in the vanguard of the field. Table 1 provides a comparative overview of state-of-the-art studies in diabetic retinopathy detection and classification, summarizing key aspects such as the dataset used, approach applied, year of publication, and key results.

**Table 1:** Comparison of state-of-the-art studies in diabetic retinopathy detection.

Reference	Year	Dataset	Approach	Key results	Plus Points
[17]	2019	Messidor and ARIA	Encoder-Decoder with Recursive Learning	The proposed OD localization method excels with 100% accuracy on Messidor and ARIA datasets, surpassing state-of-the-art methods.	Hourglass network used for OD localization. A large dataset was created to address data scarcity. High accuracy on Messidor and ARIA datasets.
[18]	2019	ORIGA and SCES	Region-Based CNN (R-CNN)	Superior performance in optic disc and cup segmentation. Enhanced accuracy in glaucoma detection.	Innovative CNN approach for joint optic disc and cup segmentation, leveraging atrous convolution and proposal networks for improved accuracy.
[19]	2017	EyePACS1	Pixel-wise Distance Regression	Precise fovea segmentation with an average error of 14 ± 7 pixels, achieved through end-to-end pixel-wise segmentation without relying on prior knowledge of other retinal structures.	Accurate fovea segmentation in retinal images using a two-stage deep learning approach with fully convolutional neural networks.
[20]	2018	Messidor	Fully Convolutional Neural Networks (CNN)	Pixelwise regression for optic disc and fovea detection, ensuring balance. Simultaneous prediction of minimal distances for joint anatomical understanding.	Simultaneous optic disc and fovea detection using effective pixelwise regression. Validation on a large dataset confirms the approach’s efficacy.
[21]	2020	ADAM and REFUGE	U-Net++ with EfficientNet Encoder	High success rates for optic disc segmentation on ADAM and REFUGE datasets. Accurate fovea detection with an average Euclidean distance of 26.17 pixels on the ADAM dataset. Top performance in OD detection and segmentation tasks in the ISBI ADAM 2020 challenge.	Simultaneous OD, cup, and fovea detection using modified U-Net++ with EfficientNet-B4. Achieved competitive performance in the ISBI ADAM 2020 challenge.
[22]	2022	A new dataset was Created: 1365 Fundus Fluorescein Angiography images with five classes.	MobileNetv2	Attained a classification accuracy of 87.40% on the collected dataset.	The new dataset, MobileNetv2, features engineering, 87.40% accuracy for diabetic retinopathy.
[23]	2022	APTOS	Pre-trained DenseNet201 with Patch Division	94.06% and 91.55% accuracy for three-class DR classification. 87.43% and 84.90% accuracy for five-class classification.	New non-fixed-size patch division model. High accuracy and robustness in DR image classification. Outperformed previous studies on the five-class APTOS 2019 dataset.
[24]	2023	ImageNet	Principal Component Analysis Multi-Label Feature Extraction	ResNet50: Accuracy of 93.67%, Hamming Loss of 0.0603 SqueezeNet1: Accuracy of 91.94%, Hamming Loss of 0.0805 ResNet152: Accuracy of 94.40%, Hamming Loss of 0.0560	Successful data pre-processing and transfer learning with ResNet50, ResNet152, and SqueezeNet1, achieving high accuracy for DR screening.
[25]	2020	EyePACS	Interpretable Classifier	Accurate classification of retina images with an interpretable model using pixel-wise score propagation for improved diagnosis insights.	A unified model for classification and interpretability with a pixel-wise score propagation approach and visual maps for ophthalmologist-friendly interpretation.
[26]	2019	Private dataset	CNN	Identification model: Sensitivity: 97.5% Specificity: 97.7% Area under the curve: 97.7% Grading model: Sensitivity: 98.1% Specificity: 98.9%	Automated DR identification and grading system achieve high sensitivity and specificity; exploration of ideal component classifiers and combinations for optimal model performance.
[27]	2021	IDRiD	Mixed Hybrid Models	Diabetic Retinopathy Detection and Classification Accuracy: 98.06% Sensitivity: 83.67% Specificity: 100%	A novel hybrid approach for DR detection and classification. High accuracy and specificity.
[28]	2022	EyePACS-1 Messidor-2 DIARETDB0	Transfer Learning and U-Net-based DR Detection	Average Accuracy: EyePACS-1: 96.60% Messidor-2: 93.95% DIARETDB0: 92.25%	Novel two-stage framework for DR classification. State-of-the-art performance on multiple datasets.
[29]	2017	DIARETDB1 MESSIDOR	SVM Hybrid Model |	Accuracy: DIARETDB1: 92.11% (Severe DME detection) MESSIDOR: 90% (Severe DME detection)	A robust method for DME detection. Provides severity grading. Tested on different datasets.
[30]	2021	IDRiD	Weighted Filters and CNN	Model precision of the Convolutional Neural Network: 0.9691	Automated diabetic retinopathy diagnosis with Gray Wolf Optimization in a deep-neural network; enhanced accuracy using Gaussian space theory and generic data structures.
[31]	2022	DIARETDB	IGWO-CNN	Classification accuracy achieved: 98.33% Outperforms other methods, including GA and GWO.	Proposed IGWO-CNN for diabetic retinopathy diagnosis. Utilized Genetic Algorithm for initial positions. Achieved 98.33% classification accuracy, outperforming other methods.
[32]	2018	MESSIDOR	Feature-based and supervised Learning	Sensitivity is comparable to ophthalmological specialists (0.9000 per patient). Specificity level of 0.6939, allowing screening of about 70% of patients with no evidence of DME.	Digital image processing for DME risk detection. Sensitivity is comparable to specialists. High specificity for patients without DME evidence.
[33]	2015	MESSIDOR	SVM	Successful texture feature extraction around the macula region for DME detection. SVM-based grading achieved promising accuracy and sensitivity.	Effective texture feature detection around the macula. Segmentation techniques for specified region extraction. Promising accuracy and Sensitivity for DME detection.
[34]	2022		DCNN	Exudate Localization	Innovative CNN-based strategy for DME classification. Emphasis on early detection in developing countries. Integration of exudates localization for enhanced diagnosis.
[35]	2021	-	3D-CNN	Binary and Multiclass Classification	A comprehensive study on data augmentation impact in CNN performance. Evaluation across binary and multiclass classification problems. Limited impact observed in architecture engineering.

## Materials and methods

This study introduces a novel method for identifying VTDR (Vision Threatening Diabetic Retinopathy) by leveraging fundus images (FIs) from the IDRiD public dataset. The approach begins with pre-processing techniques, such as FI scaling, histogram equalization, and contrast stretching, to enhance the quality of the FIs. Problems due to blurred or unclear images in the dataset necessitate these pre-processing steps. Contrast Limited Adaptive Histogram Equalization (CLAHE) helps reduce noise over-amplification by limiting contrast enhancement.

To address underfitting and overfitting concerns within the dataset, a suite of data augmentation techniques is applied to enrich and balance the data. This augmentation process includes:

- Sharpening: The images are sharpened using intensities of 0.5, 1, 1.5, and 2.
- Embossing: Applied with degrees of 0.5, 1, 1.5, and 2 for textural enhancement.
- Gaussian Blur: Implemented to smooth the images with levels of 0.25, 0.5, 1, and 2.
- Rotation: Images are rotated at specified degrees of 45, 90, 135, and 180.
- Edges Identification: Performed to outline the edges with intensities of 0.25, 0.5, 0.75, and 1.0.
- Skewing: Images are skewed in different directions, including Left, Right, Forward, and Backward.
- Flipping: Executed on the Left side, Right side, Top, and Bottom to provide different orientations.
- Shearing: Applied along the X-axis at 10Â° and Y-axis at 10Â°.

These varied and comprehensive augmentation techniques enrich the dataset, providing a more complex and diverse set of images that help to enhance the training process and improve the model’s ability to generalize across unseen data, as shown in Fig 3.

**Fig 3:** A visual representation of various augmentation procedures used to augment the FI dataset using pre-processed images.

Following pre-processing and augmentation, a unique hybrid CNN-SVD (Convolutional Neural Network-Singular Value Decomposition) model is developed to extract and select the most suitable features. The final stage involves using an enhanced SVM-RBF (Support Vector Machine-Radial Basis Function) to classify DR into five levels. The efficacy of the proposed strategy is assessed using various performance indicators such as the F1-score, accuracy, sensitivity, and specificity. The flow of this methodology is visually represented in Fig 4, delineating the organized and sequential steps adopted in this research.

**Fig 4:** Proposed methodology.

### Hierarchical block Attention-U-Net architecture

Attention mechanisms have become crucial in various computational tasks, and our innovative Hierarchical Block Attention (HBA block builds upon this growing trend. This section will delve into the details of the HBA block and the HBA-U-Net architecture, ensuring a comprehensive understanding.

### HBA block

As depicted in Fig 4, the HBA block consists of three core modules: content, relative position, and channel attention.

- Content Attention: This study formulated content attention to focus on individual pixels within each spatial feature map. This method computes an attention score between key and query vectors.
- Relative-Position Attention: This study introduced relative-position attention to encode the relative position of various retinal landmarks.
- Channel Attention: Channel-wise attention utilizes spatial information encoded into different channels in a U-Net. The approach computes the final channel attention score through specific mathematical operations.

This study designed the HBA block to scale the value vector based on content, relative position, and channel attention scores. The combined output of the HBA block employs softmax and sigmoid functions.

### HBA-U-Net architecture

The integration of HBA blocks into the U-Net without significantly increasing computational complexity led to the creation of the HBA-U-Net architecture, represented in Fig 4. It consists of:

- Encoders: These utilize ImageNet pre-trained ResNet-50 blocks to obtain feature maps at different spatial resolutions.
- Modified U-Net Structure: This structure, equipped with HBA blocks on skip connections, processes feature maps alongside the original image to produce the final fovea and OD segmentation mask.
- Incorporating HBA Blocks: The network has been re-designed to incorporate multiple HBA blocks, creating local bottleneck structures in each skip-connection pair, allowing for different spatial resolutions.

The Hierarchical Block Attention (HBA) and HBA-U-Net architecture significantly advance attention mechanisms, particularly in image segmentation. By focusing on individual pixels, spatial relationships, and channel-wise attention, this innovative model presents a refined way of processing images without drastically increasing computational requirements.

### Feature extraction and reduction using CNN-SVD

Identifying and classifying various stages of DR involves a comprehensive approach combining feature extraction and reduction to create a more streamlined and efficient model.

Initially, a Convolutional Neural Network (CNN) is utilized to extract as many Fundamental Image (FI) features as possible from the images. Using a simple CNN model, this extraction focuses on the fundamental properties that distinguish between the various DR stages. The extracted features are then processed through a series of layers involving batch normalization, max-pooling, and dropout. Batch normalization accelerates the modeling process and enhances performance by optimizing inputs, while max-pooling simplifies the data by extracting the most relevant features. Dropout, however, helps prevent overfitting, and the Adam optimizer is chosen for its robust performance with large datasets. The final dense layer of the CNN is designed to extract 256 distinct attributes from each image, each contributing to the model’s classification capabilities.

Following the extraction phase, feature reduction is employed to refine the data. This step is built on the foundational principles of the Fast Fourier Transform (FFT) method. It involves the mathematical decomposition of a matrix, represented as A of dimensions (m x n), into three distinct matrices (S, T, U) using the equation A = STU. Each of these matrices plays a specific role in transforming the data: The U matrix captures the essential structures and patterns of the image such as edges, corners, and textures; the S matrix represents the importance of each spatial feature in the image, and the T matrix reflects the singular values of the matrix.

A unique aspect of this process is using Singular Value Decomposition (SVD). By decomposing the STU matrix using SVD and selecting the top k singular values along with the corresponding left and right singular vectors, the dimensionality of the matrix is reduced. This reduction retains only the most essential features, enabling a more efficient representation. This mathematical decomposition aligns with principles such as unitary matrices and diagonal matrices, each contributing to the feature reduction process.

Overall, the combination of these two techniques, CNN for feature extraction and SVD for feature reduction, provides a powerful method to identify and classify different stages of DR. By extracting the essential elements from the images and then reducing them to their most significant characteristics, this approach streamlines the complexity of the data. It represents a balanced and sophisticated model that could offer significant advantages in diagnosing and understanding DR.


$$stu=\left[\begin{array}{cc} s_{1} & s_{2}\\ s_{3} & s_{4} \end{array}\right]\left[\begin{array}{cc} t_{1} & 0\\ 0 & t_{2} \end{array}\right]\left[\begin{array}{cc} u_{1} & u_{2}\\ u_{3} & u_{4} \end{array}\right]=\left[\begin{array}{cc} s_{1}t_{1} & s_{2}t_{2}\\ s_{3}t_{1} & s_{4}t_{2} \end{array}\right]\left[\begin{array}{cc} u_{1} & u_{2}\\ u_{3} & u_{4} \end{array}\right]=\left[\begin{array}{cc} s_{1}t_{1}u_{1}+s_{2}t_{2}u_{3} & s_{1}t_{1}u_{2}+s_{2}t_{2}u_{4}\\ s_{3}t_{1}u_{1}+s_{4}t_{2}u_{3} & s_{3}t_{1}u_{2}+s_{4}t_{2}u_{4} \end{array}\right]=t_{1}\left[\begin{array}{c} s_{1}\\ s_{3} \end{array}\right]\left[\begin{array}{cc} u_{1} & u_{2} \end{array}\right]+t_{2}\left[\begin{array}{c} s_{2}\\ s_{4} \end{array}\right]\left[\begin{array}{cc} u_{3} & u_{4} \end{array}\right]$$ (1)

Hence, PQR* can be written as:

$$\left[\begin{array}{c} |\\ S_{1}\\ | \end{array}\begin{array}{c} |\\ S_{2}\\ | \end{array}\cdots \begin{array}{c} |\\ S_{m}\\ | \end{array}\right]\left[\begin{array}{c} T_{1}\\ 0\\ | \end{array}\begin{array}{c} 0\\ T_{2}\\ | \end{array}\begin{array}{c} 0\\ 0\\ T_{m} \end{array}\right]\left[\begin{array}{c} \begin{array}{ccc} - & U_{1} & - \end{array}\\ \begin{array}{ccc} - & U_{2} & - \end{array}\\ \begin{array}{c} \vdots \\ \begin{array}{ccc} - & U_{n} & - \end{array} \end{array} \end{array}\right]=T_{1}\left[\begin{array}{c} |\\ S_{1}\\ | \end{array}\right]\left[\begin{array}{ccc} - & U_{1} & - \end{array}\right]+T_{2}\left[\begin{array}{c} |\\ S_{2}\\ | \end{array}\right]\left[\begin{array}{ccc} - & U_{2} & - \end{array}\right]+\cdots +T_{m}\left[\begin{array}{c} |\\ S_{m}\\ | \end{array}\right]\left[\begin{array}{ccc} - & U_{n} & - \end{array}\right]$$ (2)

Singular Value Decomposition (SVD) is a method that simplifies a given matrix into essential components, making it more manageable and informative. When applied to a matrix ***D***, SVD aims to find the optimal lower-rank approximation of that matrix.

Here’s a more detailed explanation of the process:

- Breaking Down the Matrix: The matrix ***D*** is divided into three distinct matrices through SVD. One of these matrices, denoted as ***T***, contains singular values that provide key insights into the structure of the original matrix.
- Selecting Higher-Valued Components: Specific values hold greater significance within the ***T*** matrix than others. These values are identified with meticulous attention to their size, and only those values beyond a preset threshold are chosen.
- Creating a Lower Rank Approximation: Constructing an optimum lower rank approximation of the original matrix ***D*** involves the selective consideration of higher-valued components from ***T***. The revised matrix preserves the essential data from the original while being condensed, enhancing its operational efficiency.
- Transforming the Matrix: The initial matrix ***D*** is thus converted into an ideal lower-rank approximation. This transformation effectively encapsulates D’s fundamental attributes while simplifying its intricacy.

Using Singular Value Decomposition (SVD) to transform a matrix into an appropriate lower-rank approximation is a very effective mathematical method. The process aids in the elimination of extraneous or less consequential data, resulting in the retention of just the most relevant elements. From a practical standpoint, this may result in enhanced computational efficiency and a more lucid understanding of the inherent patterns within the data.

### Working mechanism of novel hybrid ISVM-RBF model

The Novel Hybrid ISVM-RBF model is a flexible approach that combines an Improved Support Vector Machine with Radial Basis Function (ISVM-RBF), K-Nearest Neighbor (K-NN), and Decision Tree classifiers. This section provides an overview of the hybrid system’s fundamental concepts and operational mechanisms in relation to regression and classification tasks.The ISVM-RBF technique may be classified as a non-parametric approach, distinguishing it from traditional statistical parametric approaches. It improves the efficiency and accuracy of change detection, especially when dealing with many data samples.

- Kernel Trick: The SVM-RBF transforms variables into a high-dimensional feature space using pre-selected nonlinear mapping functions, creating a more effective classification hyperplane. This nonlinear transformation helps in both linear and nonlinear separating conditions. Radial basis functions (Gaussian variants) are the primary kernel functions used.
- Mathematical Representation: The ISVM-RBF can be represented by the following equation:

$$ISVM-RBF=\forall \omega (a,a_{i})=\exp\left(-\frac{1}{\sigma^{2}}{\left|\left|a,a_{i}\right|\right|}^{2}\right)\times \lambda$$ (3)

Characteristics and Conditions:** The SVM-RBF must meet certain symmetry and space identification conditions, as expressed in the following Eqs (4 and 5). These conditions ensure practical applicability in various real-world scenarios.


∀ω((a,p)=(φ(a).φ(p))) (4)

∀ω(a,p)−{φ(a).φ(p)}={(a).φ(p)−∀ω(a,p)} (5)

- The One vs. All binary classification technique enables data categorization into many classifications. In the context of a k-class classification issue, it is observed that each class is associated with a dedicated binary classifier, resulting in a total of k binary classifiers.

The K-nearest neighbors (KNN) algorithm is essential to this hybrid model. The classification process involves assigning items to certain categories based on the majority consensus of their k-nearest neighbors. The distances between objects are calculated using measurements like Euclidean, Manhattan, Hamming, or Minkowski.

The Decision Tree classifier partitions the data instances into homogenous subgroups using criteria such as the Chi-Square approach to measure the disparities between parent and child nodes.

Integrating these three classifiers in the Novel ISVM-RBF mixed model offers a resilient and adaptable approach for regression and classification purposes. The effectiveness of this tool in machine learning applications is attributed to its flexibility to big datasets and its capability to handle both linear and nonlinear separations.

### Performance evaluation metrics

The effectiveness of the Novel ISVM-RBF mixed model is evaluated based on many significant criteria. These measures provide a comprehensive understanding of the model’s capacity for precise prediction.

Sensitivity (True Positive Rate)

- Sensitivity is the percentage of true positives accurately classified as positives.
- A high sensitivity shows the model’s capacity to accurately identify the majority of positive instances.
- Formula:
$$Sensitivity=\frac{TP}{TP+FN}\times 100\%$$ (6)
  where TP stands for "True Positives" and FN for "False Negatives."

Specificity (True Negative Rate)

- The percentage of real negatives accurately classified as negatives is measured by specificity.
- High specificity ensures the model does not mistakenly identify negative situations as positive, which is important.
- Formula:
$$Specificity=\frac{TN}{TN+FP}\times 100\%$$ (7)

where FP represents the number of false positives, and TN represents the number of true negatives.

Accuracy

- The total percentage of accurate positive as well as negative predictions is known as accuracy.
- It comprehensively assesses the model’s performance while balancing sensitivity and specificity.
- Formula:
$$Accuracy=\frac{TP+TN}{TP+TN+FP+FN}\times 100\%$$ (8)

These performance assessment criteria provide a complete picture of the model’s advantages and disadvantages. The capacity of the model to distinguish between positive and negative examples is the focus of sensitivity and specificity. Accuracy provides a broad overview of the model’s overall performance. Lastly, the F1-Score offers an intelligent compromise between recall and accuracy, which is essential when working with unbalanced datasets. When taken as a whole, these measures provide a strong framework for comprehending and enhancing the Novel ISVM-RBF mixed model’s performance in diverse contexts.

## Results and discussion

### IDRiD dataset

This study evaluates our approach’s effectiveness through a comprehensive analysis, comparing it against prior studies conducted on the IDRiD dataset [37]. This dataset encompasses 516 retinal images, encompassing diverse pathological conditions of Diabetic Retinopathy (DR) and Diabetic Macular Edema (DME). Specifically, the dataset comprises 413 images for training purposes and an additional 103 images for testing. Notably, each image within the IDRiD dataset is accompanied by corresponding labels indicating the severity levels of DR and DME manifestations. The severity grading system classifies DR into five distinct categories, and our classification approach aligns with these five classes. For a visual depiction, Fig 5 showcases an illustrative example of fundus images alongside their respective ground truth masks. Moreover, to provide insight into the distribution of DR severity levels in the IDRiD dataset, Fig 6 displays a graphical representation. This comprehensive dataset is the foundation for evaluating and validating the proposed methodology.

**Fig 5:** (a) Fundus Images (FIs), (b) hard exudates, (c) soft exudates, (d) hemorrhages, and (e) microaneurysms.

**Fig 6:** Graphical representation of IDRiD classes distribution.

### Experimental setup

The Matlab programming environment was used for all experiments. This study used an Intel Core i7 7th generation CPU, a 1TB SSD, and 32 GB of RAM. In this section, the main outcomes of the classifier results, time complexity, and image pre-processing. In a separate presentation, the proposed work is contrasted with traditional approaches.

The hyperparameters used in the experiments played a critical role in shaping the outcomes of our study. These parameters were meticulously chosen to optimize the performance of our model. The batch size, set at 64, determines the number of training examples utilized in each iteration. A larger batch size can expedite training but may require more memory. The learning rate, specified as 0.001, influences the step size during gradient descent. A lower value ensures steadier convergence but might prolong training time, while a higher value can lead to overshooting.

Weight decay, denoted as 0.005, adds a penalty term to the loss function, encouraging smaller weight values and helping to prevent overfitting. The optimizer chosen, ADAM, is an adaptive learning rate optimization algorithm that combines the advantages of both Adagrad and RMSProp. It adapts the learning rate based on the historical gradient information, resulting in efficient convergence and reduced risk of overshooting.The loss function utilized, Categorical Cross-Entropy, measures the dissimilarity between predicted and actual class probabilities. It is well-suited for multiclass classification problems. Class weights, [–1, 1], assign different weights to different classes to address class imbalances, giving more importance to the minority class. Lastly, the number of epochs, set to 100, indicates the number of times the model iterates over the entire dataset. Too few epochs might lead to underfitting, while too many could lead to overfitting. These hyperparameters collectively dictate the training process, influencing convergence speed, model stability, and the capacity to handle imbalanced datasets.

### Image processing results

In this section, a comparison between the outcomes of pre-processing techniques and classification results. The insights drawn from Fig 4 vividly demonstrate the successful identification of illness grade 4 within the detection zones. It’s important to note that precise metrics cannot be assigned to the segmentation outcomes due to the absence of a definitive ground truth within the disease classification database.

To assess the performance of our classifiers, turn to Fig 7, which presents a comprehensive comparison. Notably, the mixed model emerges as a frontrunner in terms of performance when juxtaposed with individual models. Among the classifiers KNN, DT, SVM-P, and SVM-L, the ISVM-RBF stands out as the top performer. The consistent superiority of the Improved SVM-RBF approach across various metrics underscores this intriguing revelation. Figs 8–11 further enrich our understanding by visually portraying the enhanced predictive accuracy of the ISVM-RBF approach against alternative methodologies.

**Fig 7:** Outcomes of the classifiers.

**Fig 8:** Accuracy comparison.

**Fig 9:** Sensitivity comparison.

**Fig 10:** Specificity comparison.

**Fig 11:** Comparison of classifier performance.

In the quest for a comprehensive evaluation, consider the aspects of sensitivity and specificity, essential indicators in medical diagnostics. These nuanced comparisons are poised to illuminate the effectiveness of our proposed approach and its ability to provide robust predictions.

Based on three essential indicators, Accuracy, Sensitivity, and Specificity, Fig 12 gives a visual depiction of the performance metrics for several machine learning models, including KNN, Binary Trees, SVM-Polynomial, SVM-Linear, and Improved ISVM-RBF. On this heatmap, the x-axis shows the models, while the y-axis shows the performance data. An overview of the model’s accurate predictions concerning all other forecasts is provided by accuracy. Specificity is the percentage of genuine negatives correctly recognized, whereas sensitivity measures the proportion of real positives that are accurately detected. As a visual representation of the performance numbers, the heatmap’s color gradient, which changes from blue (poor performance) to white to red (high performance), is used. The mean performance value, normalized between 0 and 1, corresponding to the particular model and measure, is marked in each heatmap cell. The effectiveness of each model across several measures can be determined with the help of this visual tool, allowing stakeholders to make well-informed choices on model deployment or further improvement.

**Fig 12:** Confusion matrix.

Expanding on the earlier classification results, the analysis of the Receiver Operating Characteristic (ROC) curve in Fig 13 provides deeper insights into the discriminative capabilities of various classifiers. SVM-Linear, SVM-Polynomial, KNN, and Decision Tree demonstrate robust discriminatory power, boasting AUC-ROC values of 0.97, 0.98, 0.98, and 0.98, respectively. ISVM-RBF emerges as the standout performer, achieving an outstanding AUC-ROC of 0.99, highlighting its exceptional overall performance in disease classification. This higher AUC-ROC underscores ISVM-RBF’s remarkable ability to distinguish between positive and negative instances effectively, establishing it as the top-performing classifier. The ROC curve analysis, visually depicted in Fig 13, proves instrumental in assessing the trade-offs between sensitivity and specificity, aiding in selecting the most appropriate model for precise disease classification.

**Fig 13:** ROC analysis: ISVM-RBF.

### Time complexity analysis

Table 2, titled "Processing Time (PT) Complexity Analysis," comprehensively presents crucial metrics for assessing the efficiency of the image retrieval process. The total time required for each image encompasses three integral periods: pre-processing, training, and testing. This analysis highlights the intricate phases contributing to the overall processing time (PT). The pre-processing and feature extraction phase, initiating with image reading and culminating with feature extraction, is a pivotal component of the PT. Additionally, the training time accounts for the duration needed to train the entire dataset across individual classifiers. The testing time comprises the time taken for predictions and the subsequent voting process carried out by each classifier.

**Table 2:** Proposed and state-of-the-artwork comparison.

Aspect	Time Complexity (Seconds)	Additional Details
FIs Image Pre-processing and Feature Extraction	9.563562	Time taken for processing a single image, including pre-processing steps and feature extraction.
Classifier Training Time	0.437288	Time is required to train the three classifiers using the entire dataset.
Testing Time	0.037923	Time taken to test a single image using the trained classifiers.

Remarkably, this study attains a projected PT of approximately 10 seconds, a significant improvement in terms of speed. This achievement reflects the optimization achieved in both processing and computation times, enhancing the overall efficiency of the methodology. The ability to accomplish such swift processing underscores the practicality and real-time applicability of the proposed approach. This comprehensive analysis of PT intricacies deepens our understanding of the methodology’s functioning and emphasizes its potential for real-world implementation.

The presented table provides a comprehensive analysis of the Processing Time (PT) complexity and offers insights into the time required for different stages of the study. The first aspect focuses on FIs (Fundus Images) pre-processing and feature extraction, showcasing that approximately 9.56 seconds are spent on processing a single image. This includes executing various pre-processing steps and extracting relevant features contributing to the subsequent classification process.The table delves into the training time for the three employed classifiers. The training time amounts to approximately 0.44 seconds, encompassing the training of the classifiers using the complete dataset. This stage is crucial for enabling the classifiers to learn patterns and relationships within the data, enhancing their performance during testing. The testing time aspect reveals that merely 0.04 seconds are required to test a single image using the trained classifiers. This quick testing time emphasizes the efficiency of the classifiers in making accurate predictions on new, unseen data points. The concise testing process contributes to the real-time applicability of the proposed methodology. The table encapsulates the time complexities associated with different stages of the study, highlighting the efficiency and effectiveness of the proposed approach. These insights into processing and computation times offer valuable information to researchers and practitioners, aiding in understanding the practical implications and feasibility of the developed methodology.

### Comparison with state-of-the-art studies

Contextualizing the advancements made by the proposed study involves a comprehensive comparison with state-of-the-art research efforts, as depicted in Table 3. This comparison sheds light on the performance metrics achieved by various methodologies, revealing the trade-offs between accuracy and sensitivity. It is important to note that while some studies prioritize accuracy, others emphasize sensitivity, contributing to the diversity of evaluation criteria in the field. The proposed methodology stands out for its significant enhancements in accuracy and specificity. The proposed approach also achieves commendable sensitivity levels, showcasing a balanced performance across multiple evaluation dimensions.

**Table 3:** Proposed and state-of-the-artwork comparison.

Author	Year	Dataset	Method	Accuracy	Sensitivity	Specificity
[38]	2019	IDRiD	CNN+Handcrafted Features	90.70	-	-
[39]	2020	IDRiD	CANet	92.60	-	-
[40]	2020	IDRiD	CNN	90.29	88.75	96.89
		MESSIDOR		90.89	88.75	96.30
[41]	2020	IDRiD	RSNet	86.33	-	-
[42]	2020	Kaggle	CNN	81.00	-	-
[43]	2021	IDRiD	Fine KNN	94.00	-	-
		MESSIDOR		98.10	-	-
[44]	2023	IDRiD	GNN	96.00	-	-
**Proposed Work**	2023	IDRiD	ISVM-RBF	99.18	98.15	100.00

The comparison includes studies such as [38–44], each employing distinct datasets and methodologies. For instance, [35] utilized CNN combined with handcrafted features on the IDRiD dataset and achieved an accuracy of 90.70%. [40], on the other hand, employed a CNN-based approach on the IDRiD and MESSIDOR datasets, achieving accuracies of 90.29% and 90.89%, respectively, while demonstrating significant sensitivity improvements. They explored the Fine KNN method [41], achieving 94.00% and 98.1% accuracy values on the IDRiD and MESSIDOR datasets. The application of graph neural networks (GNN) by [44] resulted in an accuracy of 96.00% on the IDRiD dataset.

Importantly, the proposed study, conducted in 2023, introduces the Improved ISVM-RBF approach, yielding remarkable accuracy, sensitivity, and specificity results of 99.18%, 98.15%, and 100.00%, respectively. This advancement is underscored by a two-stage novel approach integrating U-Net models for optic disc and blood vessel segmentation, followed by the hybrid CNN-SVD model for feature extraction. Furthermore, pre-processing techniques and transfer learning contribute to the method’s efficacy. This holistic approach departs from the traditional paradigm of manually extracting features and employing conventional classifiers. The resulting improvements in diagnostic accuracy demonstrate the potential of this novel methodology in enhancing the diagnosis of Diabetic Retinopathy.

It is also important to note that the proposed methodology showcases favorable time complexity. The algorithm’s processing time is reasonable, with the most time-consuming phase being the pre-treatment technique, which takes approximately 9.5935 seconds. This efficient time profile contributes to the methodology’s potential applicability in real-world clinical settings. The presented comparison underscores the advancements made by the proposed methodology, positioning it at the forefront of the field. By effectively addressing accuracy, sensitivity, and specificity and incorporating efficient time complexity, the proposed approach offers a comprehensive and promising solution for the automated diagnosis of Diabetic Retinopathy.

### Critical analysis

The VTDR detection and classification methodology, depicted in Fig 4 and substantiated by rigorous experimentation, has delivered commendable results across multiple classifiers. The pre-processing technique, showcased in Fig 4, significantly enhances lesion accentuation, thereby improving DR detection. Two distinct algorithms contribute to lesion identification, amalgamating extracted features into a comprehensive feature vector. The introduction of a voting system, evaluated across increasing severity thresholds for each classifier, showcases impressive results. Notably, the voting system surpasses individual classifiers in classification accuracy, particularly excelling at disease severity level 4. This outcome underscores the robustness and efficacy of the approach in accurately classifying VTDR lesions.

The results are noteworthy, positioning the methodology as a frontrunner in VTDR detection and classification. A direct comparison with state-of-the-art models reveals the superior performance of the proposed hybrid CNN-SVD and ISVM-RBF models. Specifically, the ISVM-RBF model achieves an outstanding accuracy of 99.18%, sensitivity of 98.15%, and perfect specificity of 100.00%, outclassing existing benchmarks in the field.

While the methodology exhibits promising results, it is imperative to critically address the comment regarding the lack of clarity in the "Critical Analysis" section. The comprehensive evaluation includes a detailed discussion of implementation challenges: data collection, pre-processing, computing resources, hyperparameter optimization, model interpretability, and deployment considerations. These challenges are systematically analyzed to shed light on the intricacies of the methodology.

The data collection challenge emphasizes the need for a comprehensive and diverse dataset for effective model training and validation. Pre-processing complexities are highlighted, focusing on the intricate nature of retinal structures and the variability in image quality. The demand for substantial computational resources, particularly GPUs or TPUs, is recognized, specifically mentioning the proposed hybrid CNN-SVD and ISVM-RBF models.

Hyperparameter optimization emerges as a critical aspect, with a detailed acknowledgment of its time-consuming and intricate nature. The importance of achieving the optimal combination of hyperparameters for accurate lesion detection and classification is underscored. Interpretability and explainability challenges are acknowledged, emphasizing the inherent complexity of deep learning models and the need for transparent decision-making in clinical applications.

Furthermore, the deployment challenges address ethical, legal, and privacy considerations, emphasizing the need for a comprehensive framework aligned with medical standards. Overall, the critical analysis provides a comprehensive and detailed discussion of the challenges, intricacies, promising outcomes, and the superior performance of the VTDR detection and classification methodology compared to state-of-the-art models.

## Conclusion

This study underscores the transformative potential of AI in diagnosing and classifying Vision-Threatening Diabetic Retinopathy (VTDR). Leveraging a sophisticated hybrid approach that amalgamates deep learning and machine learning techniques, the proposed methodology showcases the capacity of AI to enhance VTDR identification and severity grading significantly. By integrating the strengths of multiple classifiers and a robust voting mechanism after pre-processing and feature extraction, this approach achieves an exceptional accuracy of 99.18%, 98.15% sensitivity, and 100% specificity, surpassing existing benchmarks. This substantial improvement not only underscores the proficiency of the hybrid model but also signifies a critical stride toward revolutionizing VTDR diagnosis and optimizing patient care and outcomes.

However, amidst these accomplishments, it is important to recognize the persisting multifaceted challenges. These encompass the intricacies of diverse and representative dataset collection, the meticulous nature of pre-processing procedures, the demands of substantial computational resources for training and inference, and the ethical considerations in deploying AI models within clinical settings. Ensuring model transparency and interpretability further adds to the complexity. Future endeavors could involve embracing broader and more comprehensive datasets, fine-tuning pre-processing techniques, enhancing model interpretability, and integrating advanced techniques like Generative Adversarial Networks (GANs) for data augmentation. Collaborative efforts bridging AI experts, clinicians, and regulatory bodies are crucial to shaping a future where AI-driven healthcare is at the forefront, significantly improving VTDR diagnosis accuracy and patient care strategies.
